# Human Health Activity Recognition Algorithm in Wireless Sensor Networks Based on Metric Learning

**DOI:** 10.1155/2022/4204644

**Published:** 2022-04-18

**Authors:** Dejie Sun, Jie Zhang, Shuai Zhang, Xin Li, Hangong Wang

**Affiliations:** ^1^School of Mathematics and Information Science and Technology, Hebei Normal University of Science and Technology, Qinhuangdao 066004, China; ^2^School of Information Science and Engineering (School of Software), Yanshan University, Qinhuangdao 066000, China

## Abstract

Wireless sensor network is an ad hoc network with sensing capability. Usually, a large number of sensor nodes are randomly deployed in an unreachable environment or complex area for data collection and transmission, which can realize the perception and monitoring of the target area or specific objects and transmit the obtained data to the remote end of the system. Human health activity recognition algorithm is a hot topic in the field of computer. Based on the small sample problem and the linear indivisibility of real samples encountered in metric learning, this paper proposes a human activity recognition algorithm for wireless sensor networks. Human activity recognition algorithm for wireless sensor networks uses human activity recognition algorithm to solve the singularity of intraclass divergence matrix, so as to reduce the impact of small sample problem. The algorithm maps two different feature spaces to the high-dimensional linearly separable kernel space through the corresponding kernel function, calculates the distance between samples in the two projected feature subspaces to obtain two distance measurement functions, and finally linearly combines them with weights to obtain the final distance measurement function.

## 1. Introduction

The recognition of human health activities is a hot topic in the computer field. Human activities, like language, play an important role in human communication. With the rapid development of mobile terminals, as well as the intelligent development of mobile terminals, today's mobile phones, tablets, and other devices can accurately judge simple human activities using gyroscopes and gravity sensors and send them to opposite target terminals via the network [1]. A wireless sensor network [2, 3] is a distributed network system in which a series of microsensor nodes collect and transmit data using wireless communication. Because of the characteristics and viability of this technology, this paper develops a set of human activity recognition algorithms for mobile terminals and employs wireless sensor networks to implement a series of complex commands for controlling computer terminals from mobile terminals. A wireless sensor network is a sensor-capable ad hoc network. Typically, a large number of sensor nodes are randomly deployed in environments or complex areas that are inaccessible to humans to collect and transmit data, realize perception and monitoring of target areas or specific objects, and transmit the acquired data to the system's remote end [4, 5]. For the elderly living alone, using the behavior recognition technology based on wireless sensor network to build an intelligent monitoring system indoors can not only send alarm signals in time to prevent accidents of the elderly, but also make intelligent decision-making and behavior recommendation by monitoring their daily activities [6]. For example, we can monitor the user's behavior of boiling water and then use the previous life records to find out from the data that the user has the behavior of boiling water from 8 : 00 to 9 : 00 every morning. According to this rule, we can set the electric water heater to work at 8 : 00 a.m. [7, 8].

Based on the small sample problem encountered in metric learning and the linear indivisibility of real samples, a human activity recognition algorithm for wireless sensor networks is proposed [9]. Human activity recognition algorithm for wireless sensor networks uses human activity recognition algorithm to solve the singularity of intraclass divergence matrix, so as to reduce the impact of small sample problem. The human activity recognition algorithm maps the samples from the linear nonseparable original feature space to the linearly separable high-dimensional feature space through the chi-square kernel function, then constructs the divergence matrix describing the proximity relationship between samples in the high-dimensional space, and finally obtains the projection matrix from high-dimensional to low-dimensional space by regularized linear discriminant analysis, so that the samples can still maintain the separability of high-dimensional space in low-dimensional shadow space, so as to improve the classification effect. The purpose of the method based on metric learning is to design a representation model of human activity recognition algorithm with wireless sensor networks [10, 11]. The extracted features should be robust to changes such as illumination and viewing angle and can distinguish different human activities. The most commonly used features in human activity re-recognition are color features and texture features [12, 13].

The essence of human activity recognition algorithm in wireless sensor networks based on metric learning is to learn a distance metric function through training samples, which can effectively classify samples, and make the distance between similar samples as small as possible and the distance between different samples as large as possible. Considering the difference of descriptive ability of different features, a pedestrian re-recognition algorithm based on kernel regularization linear discriminant analysis is proposed by using the idea of multifeature subspace [14]. In this algorithm, two different feature spaces are mapped to the high-dimensional linearly separable kernel space through the corresponding kernel functions, and then the projection matrices of the two feature spaces are obtained by performing regularized linear discriminant analysis in the kernel space, and the distances between samples are calculated in the two projection feature subspaces to obtain two distance measurement functions, and finally the final distance measurement function is obtained by linearly combining them with weights [15]. However, in actual research, the human activity recognition algorithm is complicated and its accuracy is low, and the effect will be even worse when processing a large amount of data, so improving recognition accuracy has become the most important task of human activity recognition at the moment. This paper focuses on a metric learning-based algorithm for human activity recognition, with the goal of learning the relationship between data using this method, making the relationship more beneficial to the recognition task, and thus improving the accuracy of human activity recognition.

## 2. Related Work

Binary sensors and motion sensors, according to [16], are used to identify ADL in the elderly. Human behavior recognition research can be divided into two categories: the first is image vision recognition, which uses image equipment to generate pictures or videos and monitor user behavior. Reference [17] employs a convolutional neural network to learn behavior data automatically using a big data analysis method to select the best features. A feature fusion method is proposed in light of the overfitting phenomenon of data labels in the learning process, which strengthens the ability of feature learning and improves the discrimination of behavior features. Although this method solves the problem of data label overfitting, it adds to the data complexity and slows down the process. Taking the video data provided by the image equipment as input, [18] proposes a moving human body segmentation algorithm based on interframe difference and an improved C-V model. The algorithm can solve the problem of recognizing moving human body behavior in complex situations and provide real-time alarms for security and monitoring systems. According to [19], wireless sensor networks have a solid business foundation as well as theoretical research significance, whether in astronomy, basic people's livelihood, or human activities. Many applications requiring the location of nodes in wireless sensor networks on a large scale, such as animal survival ecology monitoring, activity range monitoring, and so on, must solve the problem of obtaining the location of nodes in the network. Literature [20] through the big data analysis method and wireless sensor networks, with their ad hoc characteristics, further expands human vision, enables people to obtain information more safely and conveniently, enables people to explore areas unsuitable for human activities or inaccessible to human beings, and directly and efficiently obtains the information needed by human beings. The research in [21] shows that the hidden Markov model is used to segment the user's daily behavior sequence. According to the characteristics of continuity of actual actions and multisensor data fusion, a dynamic segmentation method of continuous action sequence based on hidden Markov model is proposed, and the result directly affects the accuracy of action recognition. Finally, the average recognition accuracy is 89%. This method only carries out time sequence segmentation for continuous actions and does not take into account discontinuous action sequences. Literature [22] suggests that the process of monitoring by sensors is completely transparent to users and will not affect the daily life and work of the monitored person. Sensor data is collected through a computer network and stored in a database for pattern recognition and prediction. Literature [23] proposes a design framework for data transmission scheduling and a data aggregation scheduling strategy in the network, with the goal of reducing energy consumption and data transmission delay in wireless sensor networks using big data analysis. According to [24], a wireless sensor network can transmit relevant information from the battlefield to a remote terminal without causing a network footprint due to the loss or failure of some nodes in the network, ensuring information acquisition continuity. The method of improving user behavior characteristics is presented in [25]. It proposes an algorithm for enhancing sensor data characteristics and uses the feature enhancement coefficient to express the feature recognition ability of behaviors, addressing issues such as behavior concurrency and peer diversity. Time series features are added to behavior characteristics to highlight features in the data, and the physical meaning of behavior data is improved to make it easier to understand. Although this method solves the behavior concurrency problem, it ignores the behavior similarity problem.

Based on metric learning, this paper studies the human activity recognition algorithm in wireless sensor networks. In this case, the divided time slice is used to represent the activities that occupy most of the time. However, the result is that the situation after the discretization is different from the actual situation. In order to express the difference, the discretization accuracy is introduced. When there is a rejection task, the difficulty of recognition will be increased, because it limits a part of the samples, which will make the training model unstable. Human activity recognition algorithm module is the preprocessing module of this system, which is mainly used to complete the function of human activities. It can disassemble the relationship between specific points, lines, and surfaces of human activities according to specific algorithms, and transmit these data to the calculation module.

## 3. Human Activity Recognition Algorithm Based on Metric Learning in Wireless Sensor Networks

Measurement Learning: By training and learning the wireless sensor network, we can get the appropriate Markov matrix *M*, treat the characteristics of different emotional contributions in the wireless sensor network data samples differently, and then measure the similarity of the wireless sensor network data samples more accurately, and finally achieve the goal of improving the accuracy of emotional recognition. The discretization accuracy based on metric learning indicates the percentage of correct labels in the discretized data set, and the data after discretization is used to calculate the performance metric of the model. In this paper, 1 s discrete data is used as the comparison data to evaluate the performance of the model. The algorithm of human activity recognition in wireless sensor networks based on metric learning is based on the solution set of a problem, which is called population, and there are individuals with certain gene coding properties in the solution set, and the individuals can also be considered as chromosomes. Individual chromosomes contain important information, which is expressed by a human activity recognition algorithm through gene combination. Human hair color features, for example, are determined by a gene combination of this feature. If it is to be applied to real-world problems, the first step must be coding, or expressing the characteristics of things through gene coding. A global optimization can be achieved using a human activity recognition algorithm. It differs from a general optimization algorithm in that it starts with the problem's solution set rather than a single solution at the beginning of the search. The search range is initially broad, which can serve as a good foundation for the subsequent steps and make finding the best solution easier. Metric learning is a projective space-friendly non-Euclidean metric. By finding a human activity recognition algorithm in wireless sensor networks, metric learning can reflect the fractional linear transformation of spatial structure information or semantic information of samples and model the potential relationship of training samples; it can improve discrimination. The structure of human activity recognition algorithm is given as shown in Figure 1.

The metric learning algorithm of human activity recognition algorithm draws lessons from the idea of maximum interval of SVM and learns the Markov matrix with the goal that the same sample points are as close as possible, and the different sample points are away from and maintain a large interval. It optimizes the *K* target nearest neighbors and intrusion samples of the target sample, so that the new feature space and space obtained from the original sample features are mapped. The *K* samples closest to the target sample belong to the same class, while they maintain a large interval distance from heterogeneous samples. In the process of evaluating individuals, human activity recognition algorithm only needs to calculate the fitness function value without other information. The form of fitness function can also be set for different problems, which increases the application scope of human activity recognition algorithm. In terms of recognition, clustering, and retrieval performance, although the Mahalanobis metric obtained by metric learning is better than Euclidean metric or original Mahalanobis metric, the limitations of the transformation of human activity recognition algorithm make it unable to describe the potential nonlinear relationship of training samples, which limits its application in practice. Because the expression form of the potential Riemannian manifold of the training sample is not known in advance, and the type of nonlinear transformation is also unknown, the Riemannian metric can only be approximately calculated by Euclidean metric on the training data, and the calculation efficiency is very low. In practical applications, Riemannian metric learning is not always better than Markov metric learning in recognition, clustering, and retrieval. As far as we know, there is no important breakthrough research progress in Riemannian metric learning. The framework of human activity recognition is shown in Figure 2.

The pedestrian re-recognition method based on metric learning mainly includes three stages: feature extraction, distance metric learning, and re-recognition. These advantages of human activity recognition algorithm make it widely used in parameter optimization. But its problems can not be ignored, such as nonstandard population coding, premature convergence, local optimum, and so on. In this paper, the distance measurement learning stage is studied, and the algorithm of human activity recognition is proposed. The kernel method is used to map the training samples to the linearly separable feature space, in which the divergence matrix describing the neighborhood relationship between samples is constructed, and finally a projection matrix is obtained. The flowchart analysis of human activity recognition algorithm in wireless sensor networks based on metric learning is shown in Figure 3.

The process of human activity recognition can be divided into two subprocesses: one is to extract human behavior features and fully express human behavior through feature data; the other is to construct recognition algorithm or recognition model according to the obtained features. Although the human activity recognition algorithms based on metric learning proposed in this paper have high recognition rate, in each data set with very little human activity knowledge, the kernel regularized linear discriminant analysis can not well reflect the intraclass and interclass changes of samples due to the very small number of samples in each human activity knowledge during training. Thus, the performance of the algorithm is greatly affected. Distance measurement plays a very important role in many application tasks in the field of wireless sensor network understanding and pattern recognition. The most widely used is Euclidean metric, which regards the input sample space as isotropic, so instinct has been well used.

Given a reversible symmetric matrix Ψ ∈ *R*^(*n*+1)×(*n*+1)^, its bilinear form can be represented by *ψ*(*x*, *y*).

(1) $$\begin{array}{c} \psi \left(x,y\right)=\left(x^{T},1\right)\Psi \left(\begin{array}{c} y\\ 1 \end{array}\right),\forall x,y\in R^{n}. \end{array}$$

If the matrix Ψ is positive semidefinite, let *E*^*n*^={*x* ∈ *R*^*n*^ : *ψ*_*xx*_ > 0} define

(2) $$\begin{array}{c} \rho_{E}\left(x,y\right)=\frac{k}{2_{i}}\log\left(\frac{\psi_{xy}+\sqrt{\psi_{xy}^{2}-\psi_{xx}\psi_{yy}}}{\psi_{xy}-\sqrt{\psi_{xy}^{2}-\psi_{xx}\psi_{yy}}}\right)\left(k>0\right). \end{array}$$

If the matrix Ψ is indefinite, let *B*^*n*^={*x* ∈ *R*^*n*^*|ψ*_*xx*_ < 0} define

(3) $$\begin{array}{c} \rho_{H}\left(x,y\right)=-\frac{k}{2}\log\left(\frac{\psi_{xy}+\sqrt{\psi_{xy}^{2}-\psi_{xx}\psi_{yy}}}{\psi_{xy}-\sqrt{\psi_{xy}^{2}-\psi_{xx}\psi_{yy}}}\right)\left(k>0\right). \end{array}$$

On En and Bn, *ρ*_*E*_(*x*, *y*) and *ρ*_*H*_(*x*, *y*) forces both satisfy the metric axiom, so they are metrics on En and Hn. (*R*^*n*^, *ρ*_*E*_) is called elliptic geometry space, (*B*^*n*^, *ρ*_*H*_) is called hyperbolic geometry space, *k* is a constant related to CC, 1/*k* is the curvature of elliptic geometry space, and −1/*k* is the curvature of hyperbolic geometry space. They are all special Riemann geometry, collectively called Kelley Klein metric geometry and can be unified into

(4) $$\begin{array}{c} \rho \left(x,y\right)=\frac{k}{2}\left|\log\left(\frac{\psi_{xy}+\sqrt{\psi_{xy}^{2}-\psi_{xx}\psi_{yy}}}{\psi_{xy}-\sqrt{\psi_{xy}^{2}-\psi_{xx}\psi_{yy}}}\right)\right|\left(k>0\right). \end{array}$$

The abovementioned Kelley Klein metric only depends on the symmetric matrix Ψ; that is, given a symmetric matrix, there can be a specific Kelley Klein metric.

Given a symmetric positive definite matrix *G*, its bilinear form in Kelley Klein metric can be expressed as

(5) $$\begin{array}{c} \sigma \left(x_{i},x_{j}\right)=\left(x_{i}^{T},1\right)G\left(\begin{array}{c} x_{j}\\ 1 \end{array}\right)\overset{\Delta }{=}\sigma_{ij}. \end{array}$$

Ellipse Kelley Klein measures as follows:

(6) $$\begin{array}{c} d_{ck}\left(x_{i},x_{j}\right)=\frac{k}{2i}\log\left(\frac{\sigma_{ij}+\sqrt{\sigma_{ij}^{2}-\sigma_{ij}\sigma_{ij}}}{\sigma_{ij}-\sqrt{\sigma_{ij}^{2}-\sigma_{ij}\sigma_{ij}}}\right)\left(k>0\right). \end{array}$$

The *V* support vector machine method is used as a reference in this chapter to make the Cayley-Klein metric between data points of the same class smaller and the Cayley-Klein metric between data points of different classes larger, and the following Cayley-Klein metric learning optimization model is given:

(7) $$\begin{array}{c} \min\;\sum_{i,j⟶i}\left(d_{CK}\left(x_{i},x_{j}\right)-v\beta +\mu \sum_{i}\zeta_{ijl}\right),\\ s.t.\;\left(a\right)d_{CK}\left(x_{i},x_{l}\right)-d_{CK}\left(x_{i},x_{j}\right)\geq \beta -\zeta_{ijl},\\ \left(b\right)\zeta_{ijl}\geq 0,\beta \geq 0,\\ \left(c\right)G>0, \end{array}$$

where the symbol *j*⟶*i* represents *X*_*j*_ and *X*_*i*_, which are data points belonging to the same category. The first term of the objective function punishes the large distance between the input sample and its samples of the same category, the *V* in the second term controls the proportion of misclassified sample points, the third term punishes the small distance between heterogeneous samples, and *μ* is the equilibrium constant.

With the mark *C*_*ij*_=(*x*_*i*_^*T*^, 1)^*T*^   (*x*_*j*_^*T*^, 1), there is

(8) $$\begin{array}{c} \sigma \left(x_{i},x_{j}\right)=tr\left(C_{ij}G\right)=tr\left(C_{ij}\left(L^{T}L\right)\right). \end{array}$$

In order to improve the iterative efficiency, this chapter uses small batch random gradient descent algorithm to solve the above optimization problems. Assume that the total number of samples is that, at each iteration, only *B* samples are selected to update the gradient value, where *B* is far less than the total number of samples *N*. The pedestrian re-recognition method based on metric learning needs labeled sample data in the training process to learn a metric model with good discrimination and generalization ability. However, in practical application, the cost of labeling samples is relatively high, which leads to the lack of enough training samples in metric learning and the problem of small samples.

## 4. Research on Human Activity Recognition Algorithm in Wireless Sensor Networks

### 4.1. Human Activity Recognition Algorithm for Wireless Sensor Networks Based on Metric Learning

Metric learning can be traced back to some early research. Metric learning, on the other hand, first appeared in Xing et al's 2002 proposal for the first Markov distance measurement method. It uses the nonregularized convex formula to maximize the sum of distances between points while keeping the distance between similar examples as small as possible. Some existing studies have introduced mobility into wireless sensor networks in order to maximize the network life cycle and reduce the delay in wireless sensor networks. Because rejection processing is required after measurement learning, we must manually select the rejection radius in order to achieve the same accuracy in discrimination and rejection tasks. To achieve the expected trade-off between identification and rejection tasks, the rejection radius can be selected using the cross validation method. Mobility in wireless sensor networks has a number of benefits, including improved connectivity, lower deployment costs, higher reliability, and lower energy consumption. However, using the human activity recognition algorithm, the average recognition accuracy of the human activity process is 97.42, which is 2.58 higher than the decision tree algorithm. Sensors and activity tags both use the same discrete time length, so two or more activities can happen at the same time. For example, one activity could be stopped in the middle of the time period while the other could begin right away.

Human activity recognition in wireless sensor networks based on metric learning can be divided into visual activity recognition and nonvisual activity recognition. Vision-based human activity recognition focuses on the field of computer vision, using imaging devices such as cameras and video cameras to collect information, and tracking, identifying, analyzing, and understanding activities through related processing technologies of graphics and images. Non-vision-based activity recognition mainly obtains human information through sensors such as gyroscope, gravity accelerator, and GPS. However, the feature extraction of the above methods is mostly carried out in time domain, and it is not robust compared with feature extraction in frequency domain. Another important point is that the above methods are basically based on SVM to classify different group behaviors. Human health activity recognition in wireless sensor networks can be divided into four aspects according to the complexity of the research object: posture, individual behavior, interactive behavior, and group behavior, in which interactive behavior is an action completed by two or more people, and group behavior refers to an action completed by a group of people. Measuring group behavior is influenced by complex semantics and environment, and there are relatively few studies, most of which focus on posture and individual behavior. All nodes in this architecture are static, and the receiver is mobile here. Once the receiver reaches a given sensor node and the sensor detects the existence of the receiver, data collection is completed. This architecture is beneficial to better connect to WSNs deployed in the area of interest. The process of learning human activity recognition algorithm in wireless sensor networks can usually be simplified to the classification of time-varying data; that is, the test sequence is matched with the reference sequence of typical behaviors calibrated in advance. At present, the algorithms of human behavior recognition in wireless sensor networks based on metric learning mainly include template matching method and state space method. Frame-to-frame matching method, fusion frame matching method, and key frame matching method all belong to template matching method.

### 4.2. Experimental Results and Analysis

The following is the experimental results of the measurement learning-based wireless sensor network human activity recognition algorithm model implemented in MATLAB language on the data set. This experiment adopts four algorithms, namely, decision tree algorithm, data mining algorithm, machine learning algorithm, and human activity recognition algorithm in this paper. Three experiments are carried out, as shown in Figures 4–6.

On three data sets, the recognition accuracy of the fast nearest neighbor component analysis algorithm is clearly improved when compared to the 1NN and NB algorithms, according to the experimental results. On the Weizmann data set, the average recognition accuracy of decision tree and data mining algorithms is 92.86 and 94.61, respectively, which is higher than decision tree algorithm. However, using the human activity recognition algorithm, the average recognition accuracy of the human activity process is 97.42, which is 2.58 higher than the decision tree algorithm. Sensors and activity tags both use the same discrete time length, so two or more activities can happen at the same time. For example, one activity could be stopped in the middle of the time period while the other could begin right away. The divided time slice is used to represent the activities that take up the majority of the time in this case. However, as a result of the discretization, the situation afterward differs from the actual situation. The discretization accuracy is introduced to express the difference. When a rejection task is used, the difficulty of recognition is increased because a portion of the samples is limited, making the training model unstable. In this case, however, the average recognition accuracy of the machine learning algorithm is 83.68, while the average recognition accuracy of the human activity recognition algorithm is 89.63, which is 5.45 higher than the no rejection task. Individual behavior recognition research results can be fully utilized in group behavior recognition based on individual behavior recognition. However, feature extraction in the above methods is primarily done in the time domain, which is less robust than feature extraction in the frequency domain. Another important point to note is that the methods described above use SVM to classify various group behaviors. Because SVM is difficult to apply to large samples and sensitive to missing data, metric learning is used to classify different group behaviors due to its advantages.

In this experiment, in order to evaluate the advantages and disadvantages of the human activity recognition algorithm of wireless sensor networks based on metric learning proposed in this chapter, two types of group behaviors are mainly considered, each of which is completed by individuals. The wireless sensor networks are selected, in which six segments are used as training samples and two segments are used as test samples, including frames of group target images. The group behavior corresponding to each frame is manually calibrated as a reference value. The recognition rate obtained by this method is low. The main reason is that the background is complex and the interference to recognition is large. On the other hand, only hog features are relatively single and the ability to describe behavior is limited. In general, the human activity recognition algorithm based on metric learning in wireless sensor networks has a high recognition accuracy. This experiment adopts four algorithms, namely, decision tree algorithm, data mining algorithm, machine learning algorithm, and human activity recognition algorithm in this paper. Four experiments are carried out, as shown in Figures 7–10.

The experimental results show that these methods are all based on the feature extraction of human activity recognition in wireless sensor networks based on metric learning. They need to be processed accurately in the early stage, and complex models need to be built in the later stage, which makes the whole algorithm less robust. In this paper, feature extraction in complex frequency domain can effectively suppress the influence of noise, and the whole model is simple and robust. In addition, on the sum video set, using basic methods to identify group behaviors, the recognition rates can reach 64.58% and 56.87%, respectively. Human activity recognition method based on metric learning uses linear method to classify human activity recognition samples. However, the real pedestrian sample data is often nonlinear, so it is obviously inappropriate to use linear method to solve nonlinear problems. Finally, most of the human activity recognition algorithms based on distance metric learning encounter the problem of small samples due to the lack of enough training samples. However, in this case, the average recognition accuracy of machine learning algorithm is 83.68, and that of human activity recognition algorithm is 89.63, which is 5.45 higher than that of no rejection task. Group behavior recognition based on individual behavior recognition can make full use of the existing research results of individual behavior recognition.

## 5. Conclusions

Measurement: Some existing research has introduced mobility into wireless sensor networks in order to maximize the network life cycle and reduce the delay. Because we must deal with rejection after metric learning, we must manually select the rejection radius to achieve the same accuracy in task identification and rejection. Wireless sensor networks have become increasingly popular in recent years because they are nonintrusive, private, and simple to set up. Contact switches, for example, are used to monitor how well doors and cupboards open and close. Mercury contacts are for measuring the movement of objects or the switch state of drawers. Passive infrared sensor is for detecting the movement of specific areas. The status of the flushing device is measured by a floating sensor. The human activity recognition algorithm of wireless sensor networks based on metric learning, on the other hand, uses the chi-square kernel function to map samples from the linearly indivisible original feature space to the linearly separable high-dimensional feature space, then constructs the divergence matrix describing the neighborhood relationship between samples in the high-dimensional space, and finally obtains the projection matrix from the high-dimensional space to the low-dimensional space.

## Figures and Tables

**Figure 1:** Structure diagram of human activity recognition algorithm.

**Figure 2:** Framework diagram of human activity recognition.

**Figure 3:** Flowchart of human activity recognition algorithm in wireless sensor networks based on metric learning.

**Figure 4:** Data results of different algorithms in wireless sensor networks based on metric learning.

**Figure 5:** Data results of different algorithms in wireless sensor networks based on metric learning.

**Figure 6:** Data results of different algorithms in wireless sensor networks based on metric learning.

**Figure 7:** Recognition rate of different algorithms in wireless sensor networks.

**Figure 8:** Recognition rate of different algorithms in wireless sensor networks.

**Figure 9:** Recognition rate of different algorithms in wireless sensor networks.

**Figure 10:** Recognition rate of different algorithms in wireless sensor networks.

## Data Availability

The data used to support the findings of this study are included within the article.
